The article "Supervised Computer-Aided Diagnosis (CAD) Methods for Classifying Alzheimer's Disease-Based Neurodegenerative Disorders" was retracted in 2023. Reasons: signs of a paper mill; compromised peer review; unreliable results or conclusions.

# Supervised Computer-Aided Diagnosis (CAD) Methods for Classifying Alzheimer's Disease-Based Neurodegenerative Disorders

**DOI:** 10.1155/2022/9092289

**Published:** 2022-05-23

**Authors:** Suneet Gupta, V. Saravanan, Amarendranath Choudhury, Abdullah Alqahtani, Mohamed R. Abonazel, K. Suresh Babu

**Affiliations:** ^1^Dept. of CSE, School of Engineering and Technology, Mody University, Lakshmangarh, Rajasthan 332311, India; ^2^Department of Computer Science, College of Engineering and Technology, Dambi Dollo University, Dambi Dollo, Oromia Region, Ethiopia; ^3^Department of Zoology, Patharkandi College, Karimganj-788724, Assam, India; ^4^Department of Computer Science, College of Computer Science, King Khalid University, Abha, Saudi Arabia; ^5^Department of Applied Statistics and Econometrics, Faculty of Graduate Studies for Statistical Research, Cairo University, Giza, Egypt; ^6^Department of Biochemistry, Symbiosis Medical College for Women, Symbiosis International (Deemed University), Pune, India

## Abstract

Alzheimer's disease is incurable at the moment. If it can be appropriately diagnosed, the correct treatment can postpone the patient's illness. To aid in the diagnosis of Alzheimer's disease and to minimize the time and expense associated with manual diagnosis, a machine learning technique is employed, and a transfer learning method based on 3D MRI data is proposed. Machine learning algorithms can dramatically reduce the time and effort required for human treatment of Alzheimer's disease. This approach extracts bottleneck features from the M-Net migration network and then adds a top layer to supervised training to further decrease the dimensionality and delete portions. As a consequence, the transfer network presented in this study has several advantages in terms of computational efficiency and training time savings when used as a machine learning approach for AD-assisted diagnosis. Finally, the properties of all subject slices are combined and trained in the classification layer, completing the categorization of Alzheimer's disease symptoms and standard control. The results show that this strategy has a 1.5 percentage point better classification accuracy than the one that relies exclusively on VGG16 to extract bottleneck features. This strategy could cut the time it takes for the network to learn and improve its ability to classify things. The experiment shows that the method works by using data from OASIS. A typical transfer learning network's classification accuracy is about 8% better with this method than with a typical network, and it takes about 1/60 of the time with this method.

## 1. Introduction

Alzheimer's disease (AD), the most prevalent form of illness, is a neurological disorder with an unknown cause. While AD cannot be cured with the present medical techniques [1], if properly recognized and treated, the patient's condition can be delayed. Machine learning algorithms can dramatically reduce the time and effort required for human diagnosis of Alzheimer's disease. The use of MRI signals to detect AD and NC using a machine learning transfer network is proposed in this study. The structural feature identification and time and spatial feature classification are two types of structural feature classification techniques used in MRI. The hippocampus and gray matter are primarily used to classify anatomical traits. With the rapid advancement of machine learning technology, it has been discovered that it may be employed as a quick supplemental diagnosis approach, such as modal categorization and support vector machine (SVM) algorithms. At the moment, the conventional diagnosis of AD is based on a thorough study and evaluation of clinical data by physicians, which includes the neuropsychological test of the Minimum Mental State Examination (MMSE) [2] and the electroencephalogram (EEG) of the electroencephalogram (EEG). Physiological examination [3], magnetic resonance imaging (MRI), positron emission tomography (PET), neuroimaging examination [4], and cerebrospinal fluid examination [5] are a few examples. While these procedures have produced satisfactory diagnostic findings, they are time consuming, labor expensive, and prone to some degree of subjectivity, and misinterpretation is still possible.

The article "Supervised Computer-Aided Diagnosis (CAD) Methods for Classifying Alzheimer's Disease-Based Neurodegenerative Disorders" was retracted in 2023. Reasons: signs of a paper mill; compromised peer review; unreliable results or conclusions.

When machine learning technology has been growing quickly, it has been found that it can be used as a quick auxiliary diagnosis method, such as multimodal classification [6] and support vector machine (SVM) algorithms [7]. Most of the people prefer the support vector machine because it makes significant correctness while using less computing power. It is primarily used to solve categorization challenges. The support vector machine has a memory system that is comparable to that of the SVM classifier. For big data, the SVM classification algorithm is unsuitable. MRI is a high-definition imaging technique that provides great imaging resolution, excellent contrast, and a wealth of information. It can visualize the brain's structure, reflect tiny changes, and does not emit hazardous ionizing radiation. As a result, it is now commonly utilized as an auxiliary diagnostic for AD. Classification methods for structural features in MRI may be broadly classified into structural feature classification and dimensionality reduction feature classification. The categorization of anatomical features is mostly based on the hippocampus and gray matter [8, 9].

The article "Supervised Computer-Aided Diagnosis (CAD) Methods for Classifying Alzheimer's Disease-Based Neurodegenerative Disorders" was retracted in 2023. Reasons: signs of a paper mill; compromised peer review; unreliable results or conclusions.

By contrast, dimensionality reduction feature classification only looks for features in the area of interest (ROI). It has a high rate of learning and flexible explanation skills, allowing it to represent complex features and understand nonlinear relationships. [10]. It is also possible to use MRI texture feature extraction technology [9], which is both faster and more accurate at categorization. On the other hand, the accuracy of these standard MRI machine learning techniques is based on the correctness of the features that are found. Most of them have to be manually removed, and sometimes, the process of removing features can be distressing. If the features that are extracted are wrong, the accuracy of the classification will be low. Moreover, traditional machine learning categorization is better at finding things that can be used for data mining. However, there are often some problems with picture categorization, like AD, which has characteristics that are not obvious.

In comparison with typical machine learning methods, deep learning frequently exhibits the characteristics of self-learning feature extraction for objects with uncertain features. It uses nonlinear models to transform raw data to low-level characteristics. It then abstracts high-level characteristics over numerous completely linked layers, providing more precise and efficient feature representations for categorical objects. Due to the fact that MRI is a three-dimensional (3D) picture including spatial information about brain areas, the current deep learning for AD classification is based on 3D convolutional neural networks (CNNs) [11], which can train automatically from MRI. Without segmentation of brain tissue and areas, data extraction characteristics are categorized by type. However, deep learning networks frequently require a substantial amount of training data to achieve high classification accuracy, and the amount of publically available AD MRI data remains restricted at the moment. Additionally, deep learning often involves a large number of weights combined with actual training data, which results in a lengthy training period for deep networks. Transfer learning, as a classification deep network built on tiny data, is pertained on the appropriate training dataset, minimizing the amount of time required to train on the target dataset. By bringing awareness, it is possible to reduce the formation of severe dangers and control mechanisms. Moreover, it assists in the prevention of strokes to remaining at the forefront variables. The 3D CNN approach [12, 13] was the first to employ transfer learning in MRI AD diagnosis. This method used SAE to extract features that were then applied to the network's bottom layer. In comparison, the upper layers travelled through strata that were completely linked. Accomplish. The 3D CNN may be trained and validated on the (computer-aided diagnosis of dementia, CAD Dementia) [14] dataset, as well as on the Alzheimer's Disease Neuroimaging Initiative (ADNI) dataset. The reports examines the significance of healthcare care in the distinction of Thai tourism industry products and details some of Thailand's particular medical tours customized to international markets [15].

The article "Supervised Computer-Aided Diagnosis (CAD) Methods for Classifying Alzheimer's Disease-Based Neurodegenerative Disorders" was retracted in 2023. Reasons: signs of a paper mill; compromised peer review; unreliable results or conclusions.

Although this approach achieves high classification accuracy, it does so using 3D convolution and a large number of weights. While the network files are publicly available, the pretraining weights are not, extending the training time and imposing further development constraints on the ability to grow applications. AlexNet [16] and VGG16 [17] have both been very good at diagnosing AD and so have two-dimensional transfer networks, like mobile networks. It starts with AlexNet and VGG16, then slices the MRI image, and chooses different slices depending on where they are and how much information they have. Then, the 2D convolutional neural network takes the input from the 2D convolutional network. The last categorization is done with the help of a top-level network. A slice of the MRI picture can be used as the input for a 2D convolutional neural network because the method slices it. This avoids having the 3D image and the 2D web is too different in dimension. Trimming, on the other hand, leads to the loss of information, which makes the categorization less accurate.

It comes up with a three-dimensional transfer learning network that can handle the AD and normal control (normal control, NC) classifications in MRI. It has the ability to visualize the structure of the brain, reflect minute alterations, and does not generate harmful radiation exposure. It is also beneficial to apply MRI texture feature extraction technology that is both faster and more precise. The MRI signal is a three-dimensional picture of the brain region's structure because it is high-definition imaging. We slice an MRI picture of a person into many two-dimensional pictures to start. Finally, we use supervised top-level extraction to get the top-level features of the bottleneck features. Putting the top-level parts from each slice together sends them to the network that helps classify them. When compared to other transfer learning techniques, the 3D network is able to get more feature values from MRI scans, which leads to better classification accuracy. Transfer learning is used at the same time. The bottleneck layer network is pretrained, and the top layer network is trained supervised, which significantly shortens the training time. Instead of the typical 2D transfer network, this article uses OASIS, a freely available dataset from the University of Washington's Alzheimer's Disease Research Center, and the M-Net network, which has already been trained with weights that can be downloaded. As a result, the classification accuracy goes up by about 8%, and the time it takes to do so is about 1/60 of what it takes to do with the standard stacked autoencoder (SAE) approach.

The article "Supervised Computer-Aided Diagnosis (CAD) Methods for Classifying Alzheimer's Disease-Based Neurodegenerative Disorders" was retracted in 2023. Reasons: signs of a paper mill; compromised peer review; unreliable results or conclusions.

## 2. Dimension Matching Problem

This article will use a transfer convolutional neural network for small dataset classification to classify AD because there are not a lot of public AD MRIs. To keep the classification information from being lost, a three-dimensional network-based classification method is suggested. In contrast to the previous method, the network described in this study must make sure that the data it receives has enough categorization information. At the same time, the classification network should not be too complicated, which could take a long time to train. This is the main problem with combining MRI data with transfer learning for AD classification. The MRI signal is a three-dimensional picture of the brain region's structure because it is high-definition imaging. Thus, it is a three-dimensional dataset of *MX*∗*MY*∗*MZ*, where *MX*, *MY*, and *MZ* represent the brain region's three spatial dimensions, respectively.

A frequently used technique for applying MRI data to 2D transfer learning is to break the MRI data into *MI*, 2D pictures of *M*2∗*M*3, where *Mi*, *I* = 1, 2, 3 can be *MX*, *MY*, or *MZ* to get coronal, sagittal, or axial sections. Then, these *M*1 two-dimensional slices are fed into the two-dimensional transfer network, and lastly, a top-level network is formed to accomplish the final classification. At this point, the original MRI data is reduced to 2D, resolving the 2D CNN network's input dimension problem. Because MRI is a three-dimensional (3D) image with spatial brain areas, current deep learning for AD categorization relies on 3D convolutional neural networks (CNN), which can be trained autonomously from an MRI. The efficacy of this approach, however, depends on the value of *M*1. Theoretically, the bigger the value of *N*1, the better, since it corresponds to less information lost when the original three-dimensional picture is sliced. However, because deep learning is typically a deep network, the weights increase as more ideas are input. As an example, consider a CNN network with NC convolutional layers; each convolutional layer is built of *O*1, *O*2, and *ON* feature maps with a size of *G*1∗*G*1, *G*2∗*G*2, *a*, and *GN*∗*GN*, and the convolution kernel utilized has a size of *N*1∗*N*1, *N*2∗*N*2, and *MN*∗*MN*. This is the number of weights in the network.

(1) $$\begin{array}{c} X_{\text{CNN}}=M_{1}\overset{M_{C}}{\underset{i=1}{\sum }}O_{i}\left(N_{i}N_{i}+1\right). \end{array}$$

How many weights in the network depends on how many MRI image slices *N*1 there are, so the more slices there are, the bigger it will be. Because the offset is 1, this means that this is the case rules can also be used to cut the number of parts. Among other things, one way to do this is to sort by location, with the slices closest to the brain's center being kept. If not, they are thrown away [16, 17]. A different way is to sort by picture entropy and keep the slices with the most entropy. No matter how it is cut, there will always be less information when the picture is cropped.  Figure 1 shows that the training time will be a little longer. That is why this research will look into how to balance the loss of MRI information and how complicated the transfer network is to make sure the classification network is accurate while also cutting down on how long it takes to train the network.

The article "Supervised Computer-Aided Diagnosis (CAD) Methods for Classifying Alzheimer's Disease-Based Neurodegenerative Disorders" was retracted in 2023. Reasons: signs of a paper mill; compromised peer review; unreliable results or conclusions.

## 3. Proposed Algorithms

### 3.1. The Basic Process of Classification

Use MRI data and a CNN network with transfer learning to determine if you have AD in this piece of writing. MRI is a high-resolution imaging technology that offers outstanding contrast, high imaging resolution, and a plethora of information. It has the ability to visualize the structure of the brain, reflects small changes, and does not generate harmful radiation exposure. As a result, it is now widely used as an auxiliary diagnosis for Alzheimer's disease.  Figure 2 shows how the method works in its most basic form. A network that has been trained to look for bottleneck features is used after I slice the subject's MRI data. This network looks for the bottleneck feature in each slice. When compared to traditional machine learning approaches, deep learning usually demonstrates self-learning feature extraction characteristics for objects with uncertain features. Nonlinear models are used to convert the raw data into low-level properties. Deep learning frequently uses a high number of weights in addition to actual training data, resulting in a long training period for deep networks. The bottleneck feature for each piece is then passed through the top layer to make the bottleneck feature, which makes each piece unique. It then inputs the top-level features of all slices into a classification layer to get the final classification result and finish a disease diagnosis. Accepting the top-level features is the first step. There is no need to apply different weights to each component in this training network because the weights of the bottleneck and top layers are shared across slices. Even as the number of cuts grows, the number of consequences does not get bigger. The bottleneck network for images as long as enough pieces migrate in this technique uses a 2D grid to get the characteristics of 2D slices, which makes it possible to classify 3D are made for 3D images. Simultaneously, the bottleneck layer features for each slice are extracted. The top layer of the classification network is added to the network to even more reduce the dimension by removing sections. This results in a lower feature value and easier classification network.

The article "Supervised Computer-Aided Diagnosis (CAD) Methods for Classifying Alzheimer's Disease-Based Neurodegenerative Disorders" was retracted in 2023. Reasons: signs of a paper mill; compromised peer review; unreliable results or conclusions.

## 4. Experiments

### 4.1. Experimental Setup

There is a database at the University of Washington called the OASIS database, which can be found at http://www.oasis-brains.org. The data used in this experiment comes from the OASIS-1 group. The study had 416 male and female participants who were between the ages of 18 and 96. All people, including 100 AD and 316 NC, were right-handed. Check out Table 1. In addition, each issue's downloaded data includes both the raw data and the data that has been preprocessed. The data that has been preprocessed is used as the subject of this article. The data has gone through facial features, smoothing, and correcting, normalizing, and registering, as well as other preparations [12]. Finally, in this experiment, 100 AD and 100 NC numbers were chosen, and then, the experiment was over.

### 4.2. Classification Accuracy Results

First, the accuracy of each method is shown, as shown in Table 2. There, in Table 2, the accuracy of M-Net axial 1's classification is 67.5 percent. Because this method only picks a slice that is closest to the center, the information is not complete, and the classification accuracy is not very good. The other methods in the table get categorization results by putting together many slices of a subject. Of them, the one that does not work very well at all is SAE axial 32. The rest of them work very well. The results show that using SAE to get top-level characteristics does not work very well. The results show that this strategy has a 1.5 percentage point better classification accuracy than the one that relies exclusively on VGG16 to extract bottleneck features. The use of MRI signals to detect AD and NC using a machine learning transfer network is proposed in this study. In this work, the strategy is compared to other established methodologies using MRI data from OASIS-1.

How well you can classify things has gone up by 1.5 percent with VGG16 32, 7.4 percent with M-Net 1, and 7.9 percent with the SAE axial 32 method. It also shows that the classification accuracy of a technique that uses supervised training to get top-level features and merge them at the classification layer is better than the accuracy of a technique that only uses bottleneck features.

The article "Supervised Computer-Aided Diagnosis (CAD) Methods for Classifying Alzheimer's Disease-Based Neurodegenerative Disorders" was retracted in 2023. Reasons: signs of a paper mill; compromised peer review; unreliable results or conclusions.

Figure 3 shows the graph of the feature values that the pretraining network M-Net found.  Table 3 shows the graph with the feature values. NC is the top-level feature that the pretraining network M-Net took from the NC group. AD is the top-level feature that the pretraining network M-Net took from the AD group, and so on. In the training set, there are subjects numbered 1 to 80, and in the validation set, there are subjects numbered 81 to 100. In the figure, it can be seen that most of the top-level eigenvalues of the NC group test set are between 0.8 and 1.0, while some are around 0.2 for the AD group test set.

There is a graph in Figure 4 and a table in Table 4 that shows how well each method did in the 5-time cross-validation. SAE axial 32 has better accuracy in the first and fifth experiments, but the accuracy of the rest of the tests is low, and the curve moves more. On the other hand, M-Net axial 32.

VGG16 entropy 32, these two classification methods do not have high classification accuracy in every experiment, but the fluctuations are small, so the average value is higher than the other two methods. This also shows that extracting features using the transfer learning network is better than the method of SAE.

### 4.3. Classification Time

Table 4 shows the time of extracting bottleneck features, top-level features, the time of classification layer, and each transfer method's total time. As shown in Table 5, when the number of slices is the same, the time to extract bottleneck features using M-Net (M-Net) is less than that using VGG16, which is reduced by nearly 80%. This shows that M-Net uses depthwise separable convolutions, which significantly reduces the amount of computation. It can also be seen from the table that, compared with SAE_axial_32, M-Net_axial_32 minimizes the time of extracting top-level features by nearly 96%, and the classification time is also reduced by almost 96%. The total time is reduced by almost 97%, and this all shows that under the same environment, the time to design a supervised training top layer to extract features is much less than the time to remove parts with SAE.

### 4.4. Influence of Other Factors on the Algorithm

Other parameters affecting the score of the 3D transfer learning network are discussed in this section.

To begin, the effects of each slicing method on the findings are discussed, as seen in Table 6. The slicing method is then determined by consulting the literature [16, 17], which is summarized as follows:

- The MRI scans of each person are cut axially, sagittal, and coronal. Then, 32 MRI slices in the center are chosen, including 11 axial, 11 sagittal, and 10 coronal slices
- In this step, you choose 32 axial slices for each person's MRI image slice that have the most information entropy, which is how much information there is in each slice

Third, the number of slices in the algorithm is shown, and 80, 60, 32, 20, and 10 axial slices in the center are chosen. As you can see in Table 7 and Figure 5, all other parameters of the classification algorithm are the same as in those two places.  Figure 6 shows the parameters used in the algorithm in the classification results. Tables 8 and 9 show these parameters in the figure. Overall, the number of slices that can be classified is about the same, and the development of 32 slices is a little faster than the development of the other slices. However, too many slices will make the network more complicated, and not enough slices will make the network less accurate.

The article "Supervised Computer-Aided Diagnosis (CAD) Methods for Classifying Alzheimer's Disease-Based Neurodegenerative Disorders" was retracted in 2023. Reasons: signs of a paper mill; compromised peer review; unreliable results or conclusions.

When this study is done, it talks about how different parameters of the classification layer affect how a 3D transfer network is classified. It focuses on the number of completely linked layers in the classification layer, which is important.  Table 10 shows how well Mobile Net axial 32's average classification works when there are 1, 2, 3, or 4 layers that are fully linked. Each cross-validation accuracy curve is shown in Figure 7 with Table 11. The accuracy of each curve is shown. Two completely linked layers are shown in the diagram, which shows how the categorization is put together.

The layer network has the greatest classification accuracy curve, and the table's average accuracy is the highest. Additionally, the high one is a network comprised of two fully linked layers. As a result, the design has two completely linked layers. A network with categorization layer and connection layer is a preferable choice.

This research addresses the AD classification issue for MRI data by extracting features from the slice data using the transfer learning MobileNet network. It then enters the top layer and is categorized by the classification layer network after removing the top-level characteristics. The experimental findings indicate that the approach described in this research has a higher classification accuracy than previous methods. Additionally, the running time is greatly decreased, although the following points require additional consideration.

To begin, the transfer network used in this article does not considerably increase the classification accuracy of AD when compared to the typical 3DCNN network [12, 13]. However, because 3DCNN directly inputs 3D MRI image data to the deep network, the weight will certainly rise greatly, significantly increasing the training time. The strategy described in this article exploits the 2D transfer network's pretraining significance to extract features, which dramatically reduces the pre training time. The time and classification accuracy for diagnosing AD are enhanced compared to the conventional 2D transfer network. Conventional machine learning classification is more effective at identifying items that can be exploited for data mining. However, there are frequently some issues with image categorization, such as AD, which has characteristics that are not clear. As a result, as a machine learning technique for AD-assisted diagnosis, the transfer network described in this research offers several advantages in terms of computational efficiency and training time savings. Additionally, this work employs solely MRI data to classify AD, whereas the literature [18] relies on multimodal classification approaches to achieve high classification accuracy. Along with MRI, data from PET and cerebrospinal fluid are analyzed. To improve the accuracy of the transfer network, we might look into using other types of data. Therefore, because this experiment is mostly based on data from one database, the results are limited to this database [19]. In the strict sense, more database data should be looked at to get more complete results for classification accuracy. Because this database is used by the migration network that was studied in this study, it might be easier to compare the result if this database was used. Another thing that could happen is that datasets like ADNI and CAD Dementia could be used in the future.

The article "Supervised Computer-Aided Diagnosis (CAD) Methods for Classifying Alzheimer's Disease-Based Neurodegenerative Disorders" was retracted in 2023. Reasons: signs of a paper mill; compromised peer review; unreliable results or conclusions.

Only the results of the participants' 10, 20, 32, 60, and 80 pieces are used to figure out how many slices there should be. The network does not use any other slice numbers as input. Due to the distance from the center, the slices near the two sides of the skull have less structural information [20, 21]. The more pieces, the more redundant information, and too many slices make it harder to classify and make the network run slower, so it is not considered to have more pieces [22, 23].

Only the results of the classification layer parameter setup experiment are shown. Other parameters are not looked at any more. Therefore, why is it so important to have a lot of fully linked layers? I also tried out some of the more common parts of the activation function, like Softmax, tanh, and Sigmoid. However, I found that the classification results for these functions were not very different, so the most popular ReLU was chosen [24]. The number of layer nodes that are completely linked is also important for top-level performance. It is possible to figure out how many nodes there are by looking at how many people have them. If there are not enough nodes in the network, it will not be able to handle big pictures.

On the other hand, if there are too many nodes, the training time will go up and overfitting may happen. In this article, the classification layer network has two layers that are completely linked together.

## 5. Conclusion

Using machine learning techniques to aid in identifying AD can significantly minimize the time and effort associated with human diagnosis. This article suggests the use of MRI signals to identify AD and NC using a machine learning transfer network. The transfer system proposed in this study offers significant benefits in terms of computational efficiency and training time savings as a machine learning technique for AD-assisted diagnosis. The experiment utilizes MRI data from OASIS-1, and the approach is compared to other established methods in this study. Machine learning algorithms can dramatically reduce the time and effort required for human diagnosis of Alzheimer's disease. The use of MRI signals to detect AD and NC using a machine learning transfer network is proposed in this study. The findings indicate that this technique's classification accuracy is 1.5 percentage points greater than the one that relies solely on VGG16 to extract bottleneck characteristics. Additionally, time is saved by about 80%; the accuracy is improved by approximately 8%; and overall time is saved by approximately 98 percent compared to extracting features using SAE for classification. This result demonstrates that when used with MRI data, the process of extracting top-level features from bottleneck features and then merging them at the classification layer outperforms the method of directly classifying from bottleneck features, with improved classification accuracy and less training time for supervised top-level feature training than unsupervised SAE methods.

## Figures and Tables

**Figure 1:** AD classification problem with MRI transfer learning.

**Figure 2:** Basic framework of the classification method.

**Figure 3:** Features extracted from the top layer.

**Figure 4:** Classification accuracy curves for the evaluated classification algorithms.

**Figure 5:** Accuracy of slicing methods.

**Figure 6:** Classification accuracy curves for different counts of slices.

**Figure 7:** Classification accuracy curves for different fully connected layers in a classification layer.

The article "Supervised Computer-Aided Diagnosis (CAD) Methods for Classifying Alzheimer's Disease-Based Neurodegenerative Disorders" was retracted in 2023. Reasons: signs of a paper mill; compromised peer review; unreliable results or conclusions.

**Table 1:** Parameters related to MRI data in OASIS.

Parameter	Describe	Parameter	Describe
Database	OASIS-1	Flip angle (°)	10
TR (ms)	9.7	TI (ms)	20
TE (ms)	4	TD (ms)	200

**Table 2:** Comparison of accuracy of different models.

Model	Accuracy
VGG16_entropy_32	73.4
M-Net_axial_1	67.5
SAE_axial_32	67
M-Net_axial_32	74.9

**Table 3:** features extracted from the top layer.

Serial	NC
10	10
20	15
30	20
40	25
50	26
60	27
70	28

**Table 4:** Classification accuracy curves for the evaluated classification algorithms.

Serial	VGG16_entropy_32	M-Net_axial_1	SAE_axial_32	M-Net_axial_32
1	0.65	0.64	0.7	0.8
2	0.66	0.66	0.5	0.75
3	0.67	0.65	0.55	0.7
4	0.68	0.67	0.65	0.78
5	0.7	0.68	0.8	0.9

**Table 5:** Classification algorithm running time.

Classification algorithm	Extraction bottleneck	Extract top layer	Classification layer	Total time
	Characteristic time	Characteristic time	Time	
VGG16_entropy_32	1 486.3	769.6	8.9	2 264.9
SAE_axial_32	316.1	27 304.9	161.7	27 782.7
M-Net_axial_32	309	145	7	461

**Table 6:** Comparison of accuracy of slicing methods.

Serial	M-Net_acs_32	M-Net_entropy_32	M-Net_axial_32
1	0.65	0.64	0.7
2	0.66	0.66	0.5
3	0.67	0.65	0.55
4	0.68	0.67	0.65
5	0.7	0.68	0.8

**Table 7:** Accuracy after varying slicing methods.

Classification algorithm	Accuracy
M-Net_acs_32	71
M-Net_entropy_32	72
M-Net_axial_32	74.9

**Table 8:** Classification accuracy curves for different counts of slices.

Serial	M-Net_axial_80	M-Net_axial_60	M-Net_axial_20	M-Net_axial_10	M-Net_axial_32
1	0.75	0.74	0.7	0.7	0.76
2	0.75	0.73	0.71	0.73	0.74
3	0.73	0.62	0.72	0.75	0.73
4	0.74	0.8	0.73	0.74	0.72
5	0.8	0.9	0.75	0.72	0.8

**Table 9:** Classification accuracy for various counts of slices.

Classification algorithm	Accuracy
M-Net_axial_80	72.5
M-Net_axial_60	73.5
M-Net_axial_32	74.9
M-Net_axial_20	73
M-Net_axial_10	72

**Table 10:** Classification accuracy for different fully connected layers.

Classification algorithm	Accuracy
M-Net_axial_32_one_layer	67.5
M-Net_axial_32_two_layers	74.9
M-Net_axial_32_theer_layers	71
M-Net_axial_32_four_layers	69

**Table 11:** Classification accuracy curves for different fully connected layers.

Serial	One layer	Three layers	Four layers	Two layers
1	0.65	0.66	0.8	0.6
2	0.65	0.64	0.72	0.63
3	0.63	0.63	0.72	0.65
4	0.64	0.62	0.74	0.74
5	0.7	0.7	0.75	0.72

## Data Availability

The data shall be made available on request.
